The article "Effects of Valsartan on LN, FN, MDA, Renal Tissue Fibrosis, and Inflammatory Infiltration in DN Rats" was retracted in 2023. Reasons: unreliable results or conclusions; concerns about the data; concerns about the peer review; concerns about the citations.

# Effects of Valsartan on LN, FN, MDA, Renal Tissue Fibrosis, and Inflammatory Infiltration in DN Rats

**DOI:** 10.1155/2022/6473393

**Published:** 2022-08-04

**Authors:** Yongting Qin, Gugangzhi Li, Juan Chen, Shuangli Qin, Shizhen Wang, Shanshan Chen

**Affiliations:** ^1^Department of Basic Medica, Jiangsu College of Nursing, Huaian 223005, China; ^2^Department of Endocrinology, Huai'an First People's Hospital, Huaian 223300, China

## Abstract

The effects of valsartan on laminin (LN), fibronectin (FN), malondialdehyde (MDA), renal tissue fibrosis, and inflammatory infiltration in diabetic nephropathy (DN) rats are explored. A total of 42 SPF male Sprague D (SD) rats are selected and randomly divided into normal set, model set, valsartan low-dose and high-dose sets, and metformin set with 7 rats in each set. The kidney tissue of all rats is collected after administration. The standard of protein mRNA in kidney tissues is detected by real-time fluorescence quantitative polymerase chain reaction (PCR) method, and the protein standard in kidney tissues is detected by western blot. The experimental results show that the application of valsartan to DN rats can effectively relieve the morphology of the rat kidney tissue, enhance the protein expression in the kidney tissue of the DN rats, and reduce the fibrosis and inflammatory infiltration of the kidney tissue.

## 1. Introduction

Diabetic nephropathy (DN) is the main cause of end-stage renal disease, and its pathological features are glomerular hypertrophy, mesangial thickening, glomerular basement membrane thickening, inflammatory infiltration, tissue fibrosis, etc., affecting the health of the body. At present, DN is mainly relieved by means of contrasting blood sugar and lowering blood pressure, but there is no drug for the complete therapy of DN. It is very important to find safe and effective drugs for the therapy of DN [1–3]. Valsartan is an angiotensin II receptor antagonist. As a commonly used antihypertensive drug in clinical practice, it can inhibit inflammation, reduce proteinuria in sufferers with DN, reduce podocyte damage, and has a good effect on DN. However, its effect on renal tissue fibrosis and inflammatory infiltration in DN rats is still unclear [4, 5].

This paper constructs a DN rat model to analyze the effect of valsartan on laminin (LN), fibronectin (FN), and malondialdehyde (MDA) in DN rats. A total of 42 SPF male SD rats are selected and randomly divided into normal set, model set, valsartan low-dose and high-dose sets, and metformin set with 7 rats in each set. The kidney tissue of all rats is collected after administration, and blood glucose and urine protein standards are detected. HE is used to detect the morphology of rat kidney tissues. SOD and MDA in kidney tissues are detected. The standard of protein mRNA in kidney tissues is detected by the real-time fluorescence quantitative PCR method, and the protein standard in kidney tissues is detected by western blot. The experimental results show that the application of valsartan to DN rats can effectively relieve the morphology of the rat kidney tissue, enhance the protein expression in the kidney tissue of the DN rats, and reduce the fibrosis and inflammatory infiltration of the kidney tissue.

The rest of this paper is organized as follows: Section 2 discusses related work, followed by experimental materials and methods designed in Section 3 and Section 4.  Section 5 shows the experimental results, and Section 6 concludes the paper with summary and future research directions.

## 2. Related Work

The incidence of diabetes in my country is relatively high, ranking first in the world, and with the change in the diet structure of residents, the incidence rate is increasing year by year, resulting in an increasing number of DN sufferers, abnormal glucose and lipid metabolism, proteinuria and renal fiber. Cyst is the main clinical feature of DN sufferers [6, 7]. The severe inflammatory response caused by high oxidative stress and hyperglycemia is the main pathogenic basis of DN kidney injury and fibrosis. In this examination, a rat model DN is established by intraperitoneal injection of streptozotocin. The results show that the kidney tissue of the model rats had necrosis and renal tubular epithelial cell secretion, vacuolar changes, renal tissue structural disorder and inflammation, and cell infiltration. Other pathological lesions, collagen fibers subjoined notoriously, showing obvious fibrosis and degeneration, and the expression standards of blood sugar and inflammatory factors in rats are notoriously subjoined, suggesting that streptozotocin may induce the synthesis and secretion of an extensive number of proinflammatory factors, which may cause severe inflammatory factors. Inflammation, which in turn causes abnormal glucose and lipid metabolism, proteinuria, fibrosis, and renal degeneration, indicates that the model is successfully developed [8, 9].

The main function of SOD is to scavenge free radicals in the body, while MDA is a lipid peroxidation product. Usually, if the kidney function is abnormal, the body will have a certain degree of peroxidation. SOD scavenges oxygen free radicals. If it is damaged, lipid peroxidation occurs in the body, MDA increases accordingly, and the body structure will be damaged accordingly [10, 11]. In this examination, it is found that contrast with the normal set, the model set had notoriously lower SOD and notoriously higher MDA standards (all *p* < 0.05). SOD is notoriously subjoined, MDA standard is notoriously lessened, and SOD standard is subjoined in valsartan high-dose set and metformin set, and MD standard is lessened more notoriously (both *p* < 0.05). A first-line drug, related studies have confirmed that metformin can not only reduce the blood sugar standard of the body but also can provide antioxidation to the body, inhibit the occurrence of inflammation, relieve the deposition of renal lipids, and thus protect the kidney tissue, to avoid or delay the occurrence and development of DN, so this examination used it as a positive contrast drug for DN therapy. Valsartan is a kind of antihypertensive drug. When it is applied to the therapy of DN rats, it can weaken the synthesis of inflammatory factors in the rat body to an extensive extent, avoid the further development of inflammation, and can reduce the body at the same time. The oxidative stress standard of DN is reduced, the symptoms such as proteinuria or renal fibrosis are relieved, and the development of DN is delayed [12]. LN and FN are the main components of an extensive amount of the extracellular matrix. LN and collagen together constitute the basement membrane component; FN can induce collagen formation and lead to organ fibrosis; kidney fibrosis marker gene [13]. This examination found that contrast with the normal set, the expressions of LN and FN in the model set are notoriously subjoined (all *p* < 0.05); contrast with the model set, the expressions of LN and FN in the valsartan set and metformin set are notoriously lessened. In addition, the decrease in high-dose valsartan set and metformin set is more extensive (*p* < 0.05), suggesting that valsartan may promote the normal synthesis of basement membrane, reduce the deposition of extracellular matrix, and restore normal kidney tissues [14].

As a signal transduction protein, ERK can transmit mitogen signals. It is in the cytoplasm under normal conditions and can be activated by various growth factors, peroxides, free radicals, etc., and enter the nucleus to play its role [15]. MEK is an upstream kinase of ERK and can participate in the process of ERK entry into the nucleus. The MEK-specific inhibitor U0126 can inhibit the MEK/ERK pathway and thus inhibit the migration of cavity squamous cell carcinoma [16]. Nrf1, as a mitochondrial function gene, can regulate antioxidant genes, proteasome genes, and other transcription genes, so as to play an antioxidative stress role and protect cells from oxidative stress [17]. This examination found that, in contrast with the normal set, the protein standards of MEK and p-ERK in the model set are subjoined, and the standard of Nrf1 protein is lessened (*p* < 0.05). The standard of ERK protein lessen and the standard of Nrf1 protein subjoined (*p* < 0.05); the decrease/increase is more extensive in the high-dose valsartan set and the metformin set (*p* < 0.05). Valsartan can inhibit oxidative stress, inhibit the phosphorylation expression of MEK and ERK, weaken the inhibitory effect of ERK on Nrf1, transcribe antioxidant genes, and gradually restore renal function [18]. In addition, the application of valsartan in the therapy of DN can reduce the occurrence of inflammatory reaction and avoid damage to the kidney tissue, and at the same time, the effect is enhanced with the increase of the dose. Select references [19, 20].

## 3. Experimental Materials

### 3.1. Experimental Animals

A total of 42 SPF-grade male SD rats are selected, with a body weight of 183–216 g, an average of (200.51 ± 10.33) g, and an 8-week-old animal. The animals are provided by Tianqin Biological Company. The experimental animals are temporarily raised in the animal center of Jiangsu College of Nursing. During the temporary raising period, they all had free access to water and diet and are routinely raised at a temperature of (24.5 ± 0.5)°C and (12 h/12h) (light/dark). All animal experiments are reviewed and approved by the Animal Experiment Ethics Committee of Jiangsu College of Nursing.

### 3.2. Drugs and Reagents

Valsartan capsules (specification 80 mg/capsule): National Medicine Zhunzi H20030153, were purchased from Hainan Aomeihua Pharmaceutical Co., Ltd.; metformin hydrochloride tablets (specification 0.5 g/tablet): National Medicine Zhunzi H20023370, were purchased from Sino-US Shanghai Squibb Pharmaceutical Co., Ltd.; a small animal fan, model SAR-830, was purchased from ITC, USA; an optical microscope, model CMOS, was purchased from Olympus, Japan; a multifunctional image decomposition system, model Media Cyber, was purchased from Netics, USA; a centrifuge, model LDZ5-2, was purchased from Beijing Centrifuge Factory; a microtome, model Leica electronic scale, model Metter were all purchased from Swiss CNC; a pipette, model Eppendorf, drying oven, low temperature refrigerator were all purchased from Japan Sanyo; a water bath box, medical microwave oven, were all purchased from Aidi Instrument Factory. Extracellular regulated protein kinases (ERK) (rabbit anti-mouse), primary antibody rabbit anti-mouse ERK kinase (ERK kinase, MEK), p-ERK, nuclear factor E2-related factor 1 (nuclear factor erythroid 1)-related factor, Nrf1), Lamin B1, secondary antibody goat anti-rabbit were all purchased from abcam company in the United States. A blood glucose meter was used (manufacturer: Changchun Medes Medical Equipment, model GT-1640).

### 3.3. Model Preparation and Setting

All animals are first acclimated for one week and then housed in a SPF medium. They are randomly divided into normal set, model set, valsartan low-dose and high-dose sets, and metformin set with 7 animals in each set.

Animal model preparation and set administration Reference [21]. Preparation of DN model rats: SD rats are anesthetized by intraperitoneal injection of 2.5% sodium pentobarbital solution at a dose of 45 mg/kg, the left kidney is surgically removed and fed for 1 week after suture, intraperitoneal injection of streptozotocin solution at a dose of 60 mg/kg, blood glucose is measured 72 hours later, and the results are higher than 16.7 mmol/L for at least 2 times. The model is built successfully.

### 3.4. Animal Dosing

Valsartan is dissolved in physiological saline to obtain solutions of 0.4, 0.8, and 1.6 mg/ml [22], and metformin tablets are dissolved in physiological saline to obtain a 7 mg/ml solution. The rats in the normal set and the model set are given the same dose of normal saline by gavage, once a day for 21 days.

## 4. Experimental Method

### 4.1. Sample Collection

Before the last perfusion of the experiment, the rats are fasted for 12 hours and the urine is collected for 24 hours. After the experiment, the tail vein blood is collected. The rats are killed immediately, and the kidneys are excised, some are fixed in 4% paraformaldehyde, and some are placed in a −80°C refrigerator for later use.

### 4.2. Detection of Blood Glucose and Urine Protein Standards

The fasting tail vein blood glucose standard is detected with a blood glucose meter; the 24-hour urine protein quantitative standard in the urine is detected by a 24-hour urine protein detection kit.

### 4.3. Hematoxylin-Eosin Staining (HE) to Detect Rat Kidney Tissue Morphology

The kidney tissue is taken out in 4% paraformaldehyde, sectioned (5 *μ*m in thickness), stained with hematoxylin, counterstained with ethanol and eosin, dehydrated with alcohol, cleared with xylene, mounted with neutral gum, and photographed with a light microscope. The detailed steps are sections are deparaffinized twice in xylene for 5 min each; 100%, 95%, 85%, and 70% alcohol are added within 3 min to each gradient; then, distilled water is transferred to hematoxylin stain in medium for 10 minutes; rinsed with water for about 10 s to remove excess staining solution on the incision; after rinsing with running water for 30 minutes, the core can be seen to be blue; then, it is briefly rinsed with distilled water; stained with 0.1% eosin for 5 minutes. We use 70%, 85%, 95%, and 100% dehydrated alcohol in sequence, 2  minutes for each gradient; 2 xylene washes for a total of 10 minutes; installation and sealing: we add an appropriate amount of neutral rubber and then seal it with a coverslip.

### 4.4. Detection of SOD and MDA in Kidney Tissues

A part of the kidney tissue is taken at −80°C, ground sufficiently, and the standards of SOD and MDA in the kidney are detected according to the SOD and MDA kit procedures.

### 4.5. Detection of Renal Tissue Protein mRNA by Real-Time Fluorescence Quantitative PCR

PCR detection of LN and fibronectin mRNA-NA standards. We add the TRIzol reagent to tissue cells, mix them completely, and extract total cell RNA. We select a suitable UV spectrophotometer and use it to detect the quality of total RNA at A260/A280. We choose 1 *μ*l of total RNA to dilute 50 times, add synthesize cDNA template with RNase-free dH2O, then take 10 *μ*l SYBR Green, 0.8 *μ*l forward and reverse primers, 2 *μ*l cDNA template, 0.4 *μ*l ROX Reference, add sterile water to make up to 20 *μ*l, and perform real-time PCR reaction on a fluorescent PCR instrument. The relative expression standards of LN and FN mRNA are calculated by the 2-∆∆Ct method.  Table 1 shows the PCR primer sequences.

### 4.6. Detection of Protein Standards in Kidney Tissues by Western Blot

Western blot is used to detect the protein expressions of MEK, ERK, p-ERK, and Nrf1 in the cells. The steps are as follows: collecting cells from each set, adding RIPA reagent to the cells, respectively, ultrasonicating on ice for 5 s, with an interval of 5 s, ultrasonication is done 3 times, and 4°C, and centrifuged at 12000 g for 10 min. We aspirate the supernatant solution and store at-80°C. The protein concentration is determined according to the BCA method. SDS-PAGE is performed with 5% stacking gel and 10% resolving gel. We add 30 *μ*g of protein sample to each loading well (the protein sample needs to be mixed with an equal volume of 2 × loading buffer and boiled for 5 minutes before adding to the loading well), set the voltage in the stacking gel to 80 V, and after electrophoresis is done for about 40 minutes, the blue bromophenol enters the separation gel, we set the voltage of 160 V to continue electrophoresis, and stop the electrophoresis after the bromophenol blue reaches the bottom edge. The film is transferred by a wet transfer method, the transfer voltage is set to 100 V, and the transfer time is 50 min. After transfer, the NC membrane is placed in a 5% nonfat dry milk solution and combined at room temperature for 2 h. The NC membrane is placed in the primary antibody solution and incubated at room temperature for 1 h on a shaker. The NC membrane is placed in the secondary antibody solution and combined at room temperature for 2 h. Glow with ECL. The gray value of the strip is scanned, and the relative expression standards of MEK, ERK, p-ERK, and Nrf1 are calculated according to the gray value.

### 4.7. Statistical Processing

In this examination, all the data are sorted, and a corresponding database is established for it, and all the databases are entered into SPSS 26.0 for data processing, and the measurement data are tested for normality. The multiset test is *F*, the independent samples *t*-test is used for the data between sets, and the paired samples *t*-test is used for the data within the set. *p* < 0.05, the disparity between the data is considered to be statistically extensive.

## 5. Experimental Results

### 5.1. The Expression of Glucose and Urine Protein in Different Sets of Rats

Table 2 shows the expression of glucose and urine protein in different sets of rats. In Table 2, ^*∗*^means contrast with the normal set, & means contrast with the model set, and # means contrast with the low-dose valsartan set, *p* < 0.05; the disparity is statistically extensive.  Figure 1 shows the expression of glucose and urine protein in different sets of rats. It is clearly evident from Table 2 and Figure 1 that in contrast with the normal set, the fasting blood glucose and 24 h urine protein quantification of the rats in the model set are notoriously subjoined (*p* < 0.05). It is notoriously reduced, and the reduction is more extensive in the high-dose valsartan and metformin sets, and the disparity is statistically extensive (*p* < 0.05).

### 5.2. Morphology of Kidney Tissues in Different Sets of Rats

The glomerulus and renal tubules in the normal set had clear structures and obvious shapes; in the model set, tissue fibrosis and inflammatory infiltration are obvious; in the valsartan (low, medium, and high) dose sets, tissue fibrosis and inflammatory infiltration are observed with the increase of the dose. The phenomenon gradually eased, and there is no tissue fibrosis and inflammatory infiltration of metformin.  Figure 2 shows the morphology of rat kidneys in different sets affects the results of HE staining.

### 5.3. Expression of SOD and MDA Standards in Kidney Tissues of Rats in Different Sets

Table 3 shows the expression of SOD and MDA standards in kidney tissues of rats in different sets. In Table 3, ^*∗*^ means contrast with the normal set, & means contrast with the model set, and # means contrast with the low-dose valsartan set, *p* < 0.05; the disparity is statistically extensive.  Figure 3 shows the expression of SOD and MDA standards in kidney tissues of rats in different sets. It is clearly evident from Table 3 and Figure 3 that in contrast with the normal set, the SOD of the model set is notoriously lessened, and the standard of MDA is notoriously subjoined, and the disparity is statistically extensive (all *p* < 0.05), notoriously subjoined, the standard of MDA is notoriously lessened, and the standard of SOD in the high-dose valsartan set and the metformin set subjoined, and the standard of MDA lessened more notoriously (both *p* < 0.05).

### 5.4. Contrast of LN and FN mRNA Standards in Kidney Tissues of Different Sets of Rats

Table 4 shows the contrast of LN and FN mRNA standards in kidney tissues of rats in different sets. In Table 4, ^*∗*^ means contrast with the normal set, & means contrast with the model set, and # means contrast with the low-dose valsartan set, *p* < 0.05; the disparity is statistically extensive.  Figure 4 shows the contrast of LN and FN mRNA standards in kidney tissues of rats in different sets. It is clearly evident from Table 4 and Figure 4 that in contrast with the normal set, the expressions of LN and FN in the model set are notoriously subjoined (both *p* < 0.05); contrast with the model set, the expressions of LN and FN in the valsartan set and the metformin set are notoriously lessened, and the valsartan reduction is more extensive in the high-dose set and the metformin set (*p* < 0.05).

### 5.5. Protein Standards of MEK, ERK, p-ERK, and Nrf1 in Kidney Tissues of Rats in Different Sets

Figure 5 shows the expression of MEK, ERK, p-ERK, and Nrf1 protein standards in kidney tissues of rats in different sets. In Figure 5, *A* is for the normal set, *B* is for the model set, *C* is for the valsartan low-dose set, *D* is for the valsartan medium-dose set, *E* is the for valsartan high-dose set, and *F* is for the metformin set. It is clearly evident from Figure 5 that in contrast with the normal set, the protein standards of MEK and p-ERK in the model set are subjoined (*p* < 0.05), and the protein standard of Nrf1 is lessened (*p* < 0.05). The standard of p-ERK protein lessened (*p* < 0.05), and the standard of Nrf1 protein subjoined in different dose sets of the valsartan and metformin set (*p* < 0.05). The decrease/increase is more extensive in the high-dose valsartan set and metformin set (*p* < 0.05).

## 6. Conclusion and Future Work

Valsartan can inhibit oxidative stress, thereby inhibiting the MEK/ERK signaling pathway and promoting Nrf1 expression, effectively relieving rat kidney tissue morphology, improving protein expression in kidney tissue of DN rats, and reducing renal tissue fibrosis and inflammation. Infiltration can achieve the protection of renal fibrosis, of which the high dose of valsartan has the best effect, which can be further used in clinical practice in the future.

## Figures and Tables

**Figure 1:** Expression of glucose and urine protein in different sets of rats.

**Figure 2:** The morphology of rat kidneys in different sets affects the results of HE staining: (a) normal set; (b) valsartan low-dose set; (c) valsartan medium-dose set; (d) valsartan high-dose set; (e) model set; (f) metformin set.

**Figure 3:** Expression of SOD and MDA standards in kidney tissues of rats in different sets.

**Figure 4:** Contrast of LN and FN mRNA standards in kidney tissues of rats in different sets.

**Figure 5:** Expression of MEK, ERK, p-ERK, and Nrf1 protein standards in kidney tissues of rats in different sets.

**Table 1:** PCR primer sequences.

Gene name	Base sequence
LNmRNA	upstream5′-CATGCGTGTCCGTTACAAGTG-3′
	downstream5′-CCCGTGTAGCGATTGATCTT-3′
FNmRNA	upstream5′-GGACGTACAGCTGTTATTGTG-3′
	downstream5′-TCAGCAGGAGTCACGAAGGAAT-3′

**Table 2:** Expression of glucose and urine protein in different sets of rats.

Set	Number of cases	Fasting blood sugar (mmol/L)	24-hour urine protein quantification (mg/24 h)
Normal set	7	4.69 ± 0.84	7.16 ± 1.56
Model set	7	23.18 ± 5.21^*∗*^	33.56 ± 5.57^*∗*^
Valsartan low-dose set	7	20.61 ± 3.69	26.75 ± 4.16^&^
Valsartan medium-dose set	7	16.33 ± 3.77^&^	17.66 ± 3.12^&^
Valsartan high-dose set	7	8.59 ± 1.53^&#^	9.66 ± 2.16^&#^
Metformin set	7	8.47 ± 1.66^&#^	10.33 ± 2.08^&#^

**Table 3:** Expression of SOD and MDA standards in kidney tissues of rats in different sets.

Set	Number of cases	SOD(U/ml)	MDA(*μ*mol/L)
Normal set	7	25.47 ± 6.35	34.68 ± 4.38
Model set	7	5.18 ± 1.23^*∗*^	119.36 ± 19.23^*∗*^
Valsartan low-dose set	7	8.33 ± 1.38	96.35 ± 13.19
Valsartan medium-dose set	7	13.36 ± 2.55^&^	65.17 ± 10.37^&^
Valsartan high-dose set	7	21.35 ± 2.75^&#^	42.13 ± 8.45^&#^
Metformin set	7	22.33 ± 3.16^&^	52.22 ± 9.53^&^

**Table 4:** Contrast of LN and FN mRNA standards in kidney tissues of rats in different sets.

Set	Number of cases	LN	FN
Normal set	7	1.01 ± 0.37	1.00 ± 0.21
Model set	7	2.53 ± 0.46^*∗*^	1.96 ± 0.42^*∗*^
Valsartan low-dose set	7	2.17 ± 0.49	1.85 ± 0.26
Valsartan medium-dose set	7	1.79 ± 0.45^&^	1.65 ± 0.23^&^
Valsartan high-dose set	7	1.25 ± 0.33^&#^	1.26 ± 0.16^&#^
Metformin set	7	1.31 ± 0.39^&#^	1.31 ± 0.14^&#^

## Data Availability

The simulation experiment data used to support the findings of this study are available from the corresponding author upon request.
